The article "Synthesis of Environmentally Friendly Highly Dispersed Magnetite Nanoparticles Based on Rosin Cationic Surfactants as Thin Film Coatings of Steel" was retracted in 2025. Reasons: original data or images not available; unreliable results or conclusions; concerns about the images.

# Synthesis of Environmentally Friendly Highly Dispersed Magnetite Nanoparticles Based on Rosin Cationic Surfactants as Thin Film Coatings of Steel

**DOI:** 10.3390/ijms15046974

**Published:** 2014-04-22

**Authors:** Ayman M. Atta, Gamal A. El-Mahdy, Hamad A. Al-Lohedan, Sami A. Al-Hussain

**Affiliations:** 1 Surfactant Research Chair, Chemistry Department, College of Science, King Saud University, P.O. Box-2455, Riyadh 11451, Saudi Arabia; E-Mails: khaled_00atta@yahoo.com (A.M.A.); hlohedan@ksu.edu.sa (H.A.A.-L.); imamchemistry@gmail.com (S.A.A.-H.); 2 Petroleum Application Department, Egyptian Petroleum Research Institute, Cairo 11795, Egypt; 3 Chemistry Department, Faculty of Science, Helwan University, Helwan, Cairo 11727, Egypt

**Keywords:** magnetite, nanoparticles, cationic surfactant, rosin, encapsulation, EIS, polarization

## Abstract

This work presents a new method to prepare monodisperse magnetite nanoparticles capping with new cationic surfactants based on rosin. Core/shell type magnetite nanoparticles were synthesized using *bis*-*N*-(3-levopimaric maleic acid adduct-2-hydroxy) propyl-triethyl ammonium chloride (LPMQA) as capping agent. Fourier transform infrared spectroscopy (FTIR) was employed to characterize the nanoparticles chemical structure. Transmittance electron microscopies (TEM) and X-ray powder diffraction (XRD) were used to examine the morphology of the modified magnetite nanoparticles. The magnetite dispersed aqueous acid solution was evaluated as an effective anticorrosion behavior of a hydrophobic surface on steel. The inhibition effect of magnetite nanoparticles on steel corrosion in 1 M HCl solution was investigated using potentiodynamic polarization curves and electrochemical impedance spectroscopy (EIS). Results obtained from both potentiodynamic polarisation and EIS measurements reveal that the magnetite nanoparticle is an effective inhibitor for the corrosion of steel in 1.0 M HCl solution. Polarization data show that magnetite nanoparticles behave as a mixed type inhibitor. The inhibition efficiencies obtained from potentiodynamic polarization and EIS methods are in good agreement.

## 1. Introduction

Synthesis of new bioactive materials from renewable natural resources has become a rapidly growing area to replace or partially replace environmentally and energy unfavorable toxic materials derived from petrochemicals. Rosin, a robust inexhaustible raw material from pine tree is mixture of compounds in which 90% is acidic called resin acids with the formula of C_19_H_29_COOH and the last 10% is neutral compounds. Resin acids have characteristic bulky hydrophenanetherene and two activity masses-a double-bond conjugate system and a carboxyl group that tend to participate readily in reactions that provides resin acids [1,2]. Dehydrogenated rosin and hydrogenated rosin are bioactive materials and widely used in many fields such as medicine [3,4] and antifungal activity [5]. It is well published that quaternary ammonium had robust and broad spectrum anti-fungal activity [6]. A series of Diels-Alder adducts of resin acid with acrylic acid were synthesized which had great antimicrobial activity against different kinds of bacteria by filter paper method [7,8]. As an inexpensive natural product, fungicides related to rosin have superiority. Moreover, highly active surface modified cheap rosin materials can be advantageous in the production of new materials. This is attributed to its cheap price and low toxicity when compared to the petroleum-based materials. We started to modify rosin chemical structure which can be converted to highly surface active materials to apply as additives for petroleum crude oil applications [9–18]. The corrosion protection of metals and steel has recently gained momentum using nanotechnology [19–22]. A polymer Nano composite coating can effectively protect the underlying substrate by combining the benefits of organic polymers such as water resistance and elasticity to that of advanced inorganic materials such as hardness [20]. Nanotechnology has been employed to reduce the impact of corrosive environments through the alternation of the steel/electrolyte interface (e.g., formation of Nano-composite thin film coatings on steel). Magnetite is one of the most promising nanoparticles employed in anticorrosion coatings [23,24].

Recently, magnetite (Fe_3_O_4_) nano- and micro-particles attracted more attention in material chemistry, separation technology, biology, and biomedicine, leading to a number of potential applications [25–29]. It is chemically stable, nontoxic and noncarcinogenic [30]. Many synthetic routes have been reported in the literature for chemical synthesis of these particles such as the sol-gel [31], microemulsion [32], sonochemical [33], ultrasonic spray pyrolysis [34], and microwave plasma [35]. Each preparation method has its advantages and disadvantages, which primarily relate to particles’ size distribution, production scale, and cost. Two important synthesis routes are the thermal decomposition [36] and the chemical co-precipitation reduction [37] methods. A characteristic and serious problem is in assembling and stabilizing magnetic particles as it has high affinity to agglomerate, which is an obstacle to its application and activity. This problem can be resolved if the particles are dispersed using proper dispersing agent. The surface-modification techniques that can transform these materials into valuable finished products are an important part of nanomaterials. Moreover, they allow for the manipulation of surface functions to meet diverse application requirements. Surface modification of nanomaterials with functional polymers is an important research area in polymer science owing to the wide applications. Here, we attempted to solve the synthesis of stabilized and dispersed Fe_3_O_4_ nanoparticles using chemical reduction method at ambient temperature using new cationic surfactants based on rosin as dispersing agent. Modified magnetite particles have advantages over normal organic inhibitors due to the formation of uniform thin films on the surface of steel, which entirely cover the entire surface without any defects. In the present work, it was thought valuable to investigate the application of magnetite coated with new cationic surfactants as a corrosion inhibitor for steel in an aggressive acidic medium (1 M HCl) using potentiodynamic polarization curves and electrochemical impedance spectroscopy (EIS).

## 2. Results and Discussion

### 2.1. Preparation of Cationic Surfactant

The synthetic route of LPMQA cationic surfactant was illustrated in Scheme 1. In this scheme the rosin acids was isomerized to leveopimaric acid (LPA) by heating rosin according the reported route as explained in the experimental section. The Diels Alder adduct between levopimaric acid with MA (LPMA) was reacted with oxolylchloride to produce leveopimaric chloride maleic anhydride adduct. The produced acid chloride reacted with EC in the presence of acid acceptor based on triethylamie to produce 2-hydroxy-3-leveopimaric maleic anhydride propyl chloride ester (LPME). The produced chloride ester of LLPME was reacted with TEM to produce *bis*-*N*-(3-levopimaric maleic acid adduct-2-hydroxy) propyl-triethyl ammonium chloride (LPMQA) as cationic surfactant.

IR spectra of compounds of, LPME and LPMQA are shown in Figure 1. Compared with the raw material AbA, the absorbance at 3430 cm^−1^ in the other three spectra heightens as the three-membered ring of epichlorohydrin opened and –OH is produced. The absorbance at 1700 cm^−1^ of C=O stretching vibration in spectrum of AbA converts to 1720 cm^−1^ of LPME and LPMQA after the esterification, and quaternization. The appearance of new peak around 1371 cm^−1^ was assigned to C–N stretching vibration. Due to the quaternization (Figure 1c), a small intense peak at 2365.72 cm^−1^ has appeared, which is the characteristic absorption peak of quaternary ammonium groups. The chemical structure of LPMQA surfactant was also confirmed by ^1^H NMR analysis. The spectrum of LPMQA surfactant was represented in Figure 2. The chemical shifts (δ) are 5.39 (s, 1H; OH), 4.71–4.33 (m, 2H, –CH–OH), 4.25–4.08 (m, 4H, –COO–CH_2_), 3.99–3.85 (m, 2H, –CH–OH), 3.59–3.30 (m, 16H, –CH_2_–N–), 2.50–2.37 (m, 2H), 2.22–2.10 (m, 2H), 1.95–1.39 (m, 17H), 1.38–1.24 (m, 18H, –N–CH_3_), 1.21–1.01 (m, 10H).

### 2.2. Surface Modification of Magnetite

Surface modification of nanoparticle was used to prevent agglomeration during particle synthesis by forming a dense protecting monolayer on the particle to provide effective stabilization. In the present work, we selected new cationic surfactants to stabilize the magnetite nanoparticles. The magnetite was prepared previously [38,39] at room temperature by oxidation reduction reaction of ferric chloride in the presence of potassium iodide at pH 9 using ammonia or sodium hydroxide aqueous solution and stabilized with nonionic surfactant. In the present work, the preparation and stabilization of magnetite using cationic surfactant is one of the research objectives. A schematic probable representation of the adsorption mechanism of LPMQA cationic surfactants is shown in Scheme 2. In this respect, assembling a monolayer of the LPMQA cationic surfactant molecules on the nanoparticle surface produces oil-based magnetic fluid (Scheme 2a). The aqueous-based magnetic fluid is produced by assemblies of bilayers of LPMQA surfactant molecules (Scheme 2b). The adsorption of the LPMQA cationic surfactants on the surface of Fe_3_O_4_ NPs are driven by electrostatic interactions (Scheme 2c). The charge-stabilized mechanism is most favorable to explain the interaction between magnetite surface and LPMQA cationic surfactants. The presence of LPMQA cationic surfactant, its molecules interact with the negatively charged surface of Fe_3_O_4_ NPs and create a positive surface at a pH = 9.0 via coating of the surface of Fe_3_O_4_ NPs. Therefore, at alkaline pH = 9 is found with increasing amounts of LPMQA cationic surfactant, the adsorption efficiency of the surfactant will increase on the Fe_3_O_4_ NPs surfaces. It was previously reported that [40] cetyltrimethylammonium bromide coated magnetite NPs (CTAB-coated Fe_3_O_4_ NPs) cannot interact with the positively charged Fe_3_O_4_ NPs due to electrostatic repulsion under acidic conditions. Moreover, at high concentrations of CTAB, the adsorption efficiency decreased due to the formation of CTAB (micelles and/or) ion-pairing between excess amounts of CTAB which reduce the interaction with positively charged surface of Fe_3_O_4_ NPs. Accordingly, If concentration of cationic surfactant exceeds the critical micelle concentration, micelle formation will occur. This will reduce the amount of LPMQA cationic surfactant available for particles stabilization. Attempts were made to prevent micelle formation by adding LPMQA cationic surfactant in portions. Stabilization of magnetite nanoparticles with LPMQA cationic surfactant at high pH is attributed to adsorption of LPMQA cationic ions at the particle surface and subsequent charge stabilization of the magnetic particles.

The IR spectra of pure Fe_3_O_4_ NPs and LPMQA-coated Fe_3_O_4_ NPs are shown in Figure 3. The band at 3455 cm^−1^ is attributed to the stretching vibrations of –OH, which is assigned to surface OH groups of Fe_3_O_4_ NPs (Figure 3a). The band at 571 cm^−1^ is attributed to the Fe–O band vibration of Fe_3_O_4_. Also, the band at 1380 cm^−1^ (Figure 3b) is attributed to C–N band and the peaks at 2885 and 2925 cm^−1^ are attributed to two different C–H bands vibration of LPMQA. The IR spectra show that Fe_3_O_4_ NPs surface was well modified by LPMQA. The TEM micrographs (Figure 4) of the Fe_3_O_4−_ LPMQA coated NPs demonstrate the high quality of the as-synthesized nanoparticles. The Fe_3_O_4−_ LPMQA coated NPs analyzed by TEM showed a spherical shape with a narrow size distribution (Figure 4a,b). In order to further understand the mechanism of the surfactants adsorption on the bare magnetite surface we measured the adsorption isotherm of LPMQA rosin surfactants on the hydrophilic magnetite particles in water as illustrated in the experimental section. The absorbance values of the absorbed LPMQA on the magnetite were determined *vs.* concentrations and plotted to fit the equation *Y* = *a* + *bX*; where *Y* represents the absorbance and *X* is the concentration of the surfactants. The equations (with *r*^2^ = 0.9997) were obtained as absorbance = 0.001 + 0.163 *C*. The adsorption activity of LPMQA on the surface of hydrophilic magnetite was measured and listed in Table 1. The data show that the adsorbed amounts at LPMQA displays two plateaus. The first at low concentrations corresponds to the interaction between cationic nitrogen groups and hydroxyl groups of the magnetite as illustrated in Figure 3. It is thus suggested that the initial adsorption of LPMQA molecules on the particles is driven by electrostatic interaction. Increasing the concentration of LPMQA increases monotonously just before the second plateau is reached at 1.9 mM which was determined as the optimum concentration of LPMQA surfactant to adsorb onto the dispersed bare magnetite nanoparticles (concentration 10%). It is suggested that the LPMQA molecules form a monolayer on the particle surface with their hydrocarbon chains towards water, *i.e.*, the adsorption is via the interaction of the LPMQA nitrogen head groups with the OH of magnetite surface. These results indicated that the LPMQA rosin surfactant molecules first adsorb as individual molecules through interaction with OH groups of magnetite, and then associate into hemimicelles. In the hemimicelles, the surfactants attach their head-groups to the magnetite surface and orient their tail groups toward solution, thus forming hydrophobic patches on the surface [41]. Further adsorption then brings an increasing number of surfactants to the interface to form a complete second layer of bilayer on magnetite surfaces [41].

The image reveals the formation of monodisperse nanoparticles with an average size of 12.5 nm confirming that the proposed scheme is an effective method for the preparation of monodisperse magnetic nanoparticles. The magnetite nanoparticles appear as spherical dots with very narrow size distributions, typically 5%–10%. The spontaneously formed ordered assembly pattern is an additional confirmation of the monodispersity of the nanoparticles. The thickness of the shells is 3.7 nm. The thickness of the surfactant shell estimated using the difference between the magnetite core and the thickness of coated magnetite core shell as illustrated in the high resolution TEM micrograph at the bottom of Figure 4a.

Figure 5 shows the XRD pattern of the synthesized NPs, which is quite identical to pure magnetite (JCPDS No. 07-0322), indicating that the sample has a cubic crystal system. Also, it can be seen that no characteristic peaks of impurities were observed which demonstrates that the designed reaction procedure is effective to synthesize pure Fe_3_O_4_ NPs. The calculated d-spacing, matches well to the major d-spacing of magnetite (Fe_3_O_4_) [42,43]. The average size of the magnetite nanoparticles was estimated as 11.7 nm using the Scherrer equation: *d* = 0.9 λ/Δ(2θ)cosθ, where *d* is the crystalline domain size, Δ(2θ) is the width at half-maximum of the strongest peak (311), and λ is the X-ray wavelength. The Fe_3_O_4_ NPs size is in good agreement with the average diameter measured from TEM (12.5 nm).

### 2.3. Potentiodynamic Polarization

The potentiodynamic polarization curves for corrosion of steel in 1 M HCl, solutions without and with magnetic nanparticles were shown in Figure 6. The presence of magnetic nanparticles causes a prominent shift for both anodic and cathodic curves to lower values of current densities. The anodic and cathodic reactions of steel are clearly inhibited with increasing the concentration of magnetic nanparticles. This result suggests that addition of magnetic nanparticles in 1 M HCl solutions significantly reduces anodic dissolution and retards the cathodic reaction of steel. The results clearly indicate that magnetic nanparticles act essentially as a mixed type inhibitor in 1 M HCl solutions. The inhibition action is caused by geometric blocking effect by a reduction of the active sites area on the surface of the corroding steel [44]. It can be concluded that both cathodic and anodic reactions of steel corrosion are drastically retarded by the addition of magnetic nanparticles in 1 M HCl solutions. Accordingly, the corrosion current density values are estimated accurately by extrapolating the cathodic and anodic linear region to the corrosion potential. The electrochemical corrosion parameters including corrosion current densities (*i_corr_*), corrosion potential (*E_corr_*), anododic Tafel slope (*Ba*), cathodic Tafel slope (*Bc*) and corresponding inhibition efficiency (*IE*%) are given in Table 2. The inhibition efficiency (*IE*%) was calculated from potentiodynamic polarization using the following relationship [45–47]:

(1) $$IE\%=1-i_{corr\;(inh)}/i_{corr\;(uninh)}\times 100$$

where *i_corr (uninh)_* and *i_corr (inh)_* are corrosion current density values in the absence and presence of inhibitor, respectively. The inhibition efficiencies (*IE*%) were also listed in Table 2. It is evident that *IE*% increases with the inhibitor concentration, due to an increase in the blocked area of active sites of the steel surface. The decrease of corrosion rate may be explained by the inhibitory action of inhibitor on cathodic and anodic branches of the polarization curves by blocking the anodic and cathodic active sites on the steel surface.

### 2.4. Electrochemical Impedance Spectroscopy (EIS)

Figure 7 shows the typical Nyquist diagram for corrosion of steel in 1 M HCl solution with and without inhibitor. The impedance diagrams consist of single semicircle capacitive loop indicating a charge-transfer process mainly controlling the corrosion of steel. The EIS plots can be interpreted by an equivalent circuit with a solution resistance (*Rs*), a charge transfer resistance (*Rct*) and a double layer capacitance (*Cdl*) as shown in Figure 8. The circuit employed allows the identification of both charge transfer resistance (*Rct*) and double layer capacitance (*Cdl*). The fit parameters were analyzed using Zview2 software and listed in Table 1. The inhibition efficiencies (*IE%*) for the corrosion of steel were calculated and also listed in Table 1 by means of the following equation [45–47]:

(2) $$IE\%=1-R^{\circ }ct/Rct_{\left(inh\right)}$$

where *R*°*ct* and *Rct_(inh)_* are the values of the charge transfer resistance without and with inhibitor, respectively. As can be seen from the data presented in Table 2, the inhibition efficiencies increase significantly with the concentration of inhibitor. It can be concluded that magnetic nanoparticles exhibit effective inhibition for the corrosion of steel in 1 M HCl solution. As the inhibitor concentration increased, the *Rct* values increased, but the *Cdl* values tended to decrease. The decrease in *Cdl* value may be accounted to the adsorption of inhibitor on steel surface, which led to an increase in *IE%* [48–50]. In addition, the decrease in the *Cdl* values can be attributed to a decrease in local dielectric constant and/or an increase in the thickness of the electrical double layer, which enhance the adsorption of inhibitor on the steel surface. The inhibition efficiencies, calculated from potentiodynamic polarization curve and EIS measurements are in reasonably good agreement. The results of EIS and polarization measurements are in good agreement with that reported previously for improving the anticorrosive performance of steel with the addition of nanoparticles to corrosive medium [51–53].

## 3. Experimental Section

### 3.1. Materials

Gum rosin was obtained from Wuzhou Chemical, China and used as received. Rosin acid (AbA) with acid number 165 mg KOH·g^−1^ was obtained from a commercial resin by crystallization from cooled concentrated acetone solutions and purified by recrystallization from the same solvent. The separation of the resin acids from rosin was carried out to increase the yield and to remove terpens. Maleic anhydride (MA), epichlorohydrin (EC), tetrahydrofuran (THF), acetate acid, triethylamie (TEA) and oxalyl chloride (C_2_Cl_2_O_2_) were purchased from Aldrich Chemical Co. Anhydrous ferric chloride (St. Louis, MO, USA) potassium iodide and aqueous (25%) ammonium hydroxide solution used as reagents for preparation of magnetite were purchased from Aldrich Chemical Co. (St. Louis, MO, USA). Leveopimaric maleic anhydride adduct (LPMA) was prepared as reported in the previous work [18].

### 3.2. Preparation Methods

#### 3.2.1. Synthesis of *Bis-N*-(3-levopimaric maleic acid adduct-2-hydroxy) Propyl-Triethyl Ammonium Chloride (LPMQA)

LPMA (10 g, 0.025 mol) was dissolved in 50 mL THF and added to a round bottom flask. Oxalyl chloride (2.95 mL, 0.03 mol) was injected and stirred at 50 °C for 4 h. The gas generated in the reaction was absorbed by base solution. After removed of the unreacted oxalyl chloride by vacuum distillation, the LPMA chloride (LPCMA) was obtained. Then, epichlorohydrin (18.5 g, 0.2 mol) and TEA (0.32 g, 0.001 mol) were added dropwise and the reaction temperature was heated to 50 °C and kept for 4 h. A high viscosity liquid was obtained after reduced pressure distillation was used to remove the excess epichlorohydrin. Then the mixture was extracted by ether and water three times. Aqueous phase remained and distilled under reduced pressure for recrystallization from alcohol and acetone. The produced *bis-N*-(3-levopimaric maleic acid adduct-2-hydroxy) propyl-triethyl ammonium chloride (LPMQA) was obtained as light yellow powder has yield: 72%.

#### 3.2.2. Preparation of Modified Magnetite Nanoparticles

The modified magnetite nanoparticles were made by coating magnetite with LPMQA. In this respect, a solution of anhydrous FeCl_3_ (40 g) in distilled water (300 mL) was prepared and named aqueous solution A. Further, potassium iodide (13.2 g, 0.08 mol) was dissolved in distilled water (50 mL) to prepare an aqueous solution B. The aqueous solutions A and B are then mixed together at room temperature, stirred and allowed to reach equilibrium for one hour while bubbling with pure N_2_ to keep the mixture oxygen free throughout the preparation procedure. LPMQA (3 g) diluted in water (100 mL) was added after heating the reaction mixture at 40 °C under vigorous stirring, then NH_4_OH (25%, 200 mL) was added dropwise to the above solution. After that, the reaction mixture was stirred for another 0.5 h at 50 °C. Finally, the LPMQA-stabilized Fe_3_O_4_ nanoparticles were separated from the mixture by ultracentrifugation at 12,000 rpm, washed with water three times and with ethanol two times.

### 3.3. Characterization

Fourier Transform infrared (FTIR) spectroscopic analysis of the samples was performed using a Spectrum One FTIR spectrometer (Perkin-Bhaskar-Elmer Co., Boston, MA, USA).

^1^H NMR (400 MHz Bruker Avance DRX-400 spectrometer; (Bruker Analytische Messtechnik, Karlsruhe, Germany) was used to investigate the chemical structures of the prepared rosin derivatives using CDCl_3_ as solvent and tetramethylsilane (TMS) as an internal reference. The morphology and structure of the prepared magnetic nanoparticles were determined using high-resolution transmission electron microscopy (HR-TEM). HR-TEM images of the nanocomposites were recorded using a JEM-2100 F (JEOL, Tokyo, Japan) at an acceleration voltage of 150 kV. The particle size distributions (PSDs) were determined from TEM microphotographs on representative samples of more than 1000 particles of magnetic latexes and analyzed using the Bolero software (AQ Systems, Tyresö, Sweden). A magnetite nanoparticle solution (1 mg) was diluted into 10 mL of ethanol, sonicated for 5 min and the resulting magnetite dispersed solutions solution. A few drops of the magnetite dispersed in ethanol solution were placed onto a carbon coated copper grid and allowed to evaporate. XRD patterns of the samples were obtained using a diffractometer (MiniFlex X-ray diffractometer/PW 3710, Rigaku, Japan) equipped with Cu–Ka (λ = 0.154 nm) radiation.

### 3.4. Materials

The experiments were performed with steel specimens with the following chemical composition (wt %): 0.14% C, 0.57% Mn, 0.21% P, 0.15% S, 0.37% Si, 0.06% V, 0.03% Ni, 0.03% Cr and the remainder Fe. Prior to experiments, the specimens were successively polished using emery papers from 100 to 4000 grade. Then, the specimens were washed with distilled water and degreased with acetone and dried with a cold air.

### 3.5. Measurement of Adsorption Isotherm of LPMQA on Magnetite Nanoparticles

Bare magnetite particles (0.3 g; 2 wt %) were dispersed in 15 mL of double distilled water containing different concentrations of the prepared surfactants (ranged from 0.1–5 wt %) using an ultrasound probe for 2 min at 50 W output and the dispersions were put in a thermostatic chamber at 25 °C for 10 min. The suspended particles were separated by centrifugation (8000 rpm for 10 min), the concentration of the prepared surfactants in the supernatant was measured using a spectrophotometric method. This could be achieved by monitoring the intensity of the absorption at 285 nm. A calibration curve (based on Beer’s low) represents the variation of rosin surfactant absorbance *vs.* their concentrations. The absorbance values of the rosin blank solutions in the absence of silica were determined as blank absorbance. The concentration of the absorbed surfactants on magnetite particles was determined from absorbance differences between blank solution and surfactant concentrations in the supernatant (after separation of silica by centrifuge). The adsorption activity values can be calculated as; activity = [(*C*_o_ − *C*) × 100/(*C*_o_)] where; *C* and *C*_o_ are concentrations of rosin surfactants (mmol/L) in the presence and absence of magnetite particles, respectively.

### 3.6. Electrochemical Measurements

A three-electrode system including a steel as working electrode (WE), Pt sheet as counter electrode (CE) and saturated calomel electrode (SCE) as a reference electrode (RE) were used for electrochemical measurement. Potentiodynamics polarization measurements were conducted with a computer-controlled (potentiostat/galvanostat) Solartron 1470E system (Solartron Analytical, Cambridge, UK). Impedance measurements were carried out using Solartron 1470E system (potentiostat/galvanostat) with Solartron 1455A (Solartron Analytical, Cambridge, UK) as frequency response analyzer in the frequency range of 10 mHz–100 kHz using a 10 mV peak-to-peak voltage excitation. Data were collected and analyzed using CorrView, Corr-Ware, Zplot and ZView software (Scribner Associates Inc., Cambridge, UK).

## 4. Conclusions

1. Rosin quaternary ammonium salt derivative LPMQA was synthesized by three steps in this work. The structure of target products was characterized by IR, ^1^H NMR.
2. The data indicated that the LPMQA cationic surfactant was chemically adsorbed at the magnetite surfaces. The charge-stabilized mechanism is most favorable to explain the interaction between magnetite surface and LPMQA cationic surfactants.
3. The formation of monodisperse nanoparticles with an average size of 12.5 nm confirms that the proposed scheme is an effective method for the preparation of monodisperse magnetic nanoparticles. The Fe_3_O_4_ NPs size is in good agreement with the average diameter measured from TEM (12.5 nm).
4. Magnetic nanoparticles were an effective inhibitor for corrosion of steel in 1 M HCl solution and the inhibition efficiency increased with increasing concentration. The inhibition efficiencies, calculated from potentiodynamic polarization curve and EIS measurements are in reasonably good agreement.
5. Magnetic nanoparticles inhibit the corrosion of steel by controlling both anodic and cathodic reactions in 1 M HCl solution and acts as a mixed type inhibitor.

## Figures and Tables

**Figure 1.** FTIR spectra of: (a) rosin AbA; (b) LPME; (c) LPMQA.

**Figure 2.** ^1^H NMR spectrum of LPMQA.

**Figure 3.** FTIR of spectra of: (**a**) pure Fe_3_O_4_ NPs; and (**b**) Fe_3_O_4_ NPs coated with LPMQA.

**Figure 4.** TEM micrograph (**a**) and histogram (**b**) of the as-prepared magnetite nanocrystals. The *y*-axis of the histogram represents the number of particles.

**Figure 5.** XRD pattern of the synthesized (**a**) bare Fe_3_O_4_ NPs; and (**b**) Fe_3_O_4_coated with LPMQA.

**Figure 6.** Potentiodynamic polarisation curves for steel in 1.0 M HCl without and with different concentrations of inhibitor.

**Figure 7.** Nyquist plot for steel in 1.0 M HCl without and with different concentrations of inhibitor.

**Figure 8.** Equivalent circuit used to fit EIS data.

**Scheme 1.** Synthetic routs of LPMQA.

**Scheme 2.** Schematic illustration of the adsorption mechanism of (**a**) monolayer assembly; (**b**) double layer assembly and (**c**) chemical interaction of LPMQA onto Fe_3_O_4_ NPs.

**Table 1.** Adsorption of the LPMQA prepared surfactants on the surface of the dispersed magnetite particle (10 wt %).

Surfactant Concentrations		Adsorption Activity (%)

wt %	mol/L	
0.288	0.0048	36.4
2.88	0.048	38.3
5.76	0.096	48.3

**Table 2.** Inhibition efficiency values for steel in 1 M HCl with different concentrations of inhibitor calculated by Polarization and Electrochemical Impedance Spectroscopy (EIS) methods at 25 °C.

Polarization Method						EIS Method		
	
	*Ba* (mV)	*Bc* (mV)	*E_corr_* (V)	*i_corr_* (μA/cm^2^)	*IE*%	*Rct* (Ohm)	*Cdl* (μF/cm^2^)	*IE*%
Blank	147.00	141.00	−0.4034	745	-	1.80	334	-
50 ppm	93.63	128.85	−0.4050	191.17	74.34	6.90	189	73.91
150	112.70	147.85	−0.4156	167.8	77.40	8.07	152	77.89
250	113.53	113.00	−0.4496	89.40	88.00	15.01	136	88.00
